# Application of 24 h Dynamic Electrocardiography in the Diagnosis of Asymptomatic Myocardial Ischemia with Arrhythmia in Elderly Patients with Coronary Heart Disease

**DOI:** 10.1155/2022/3228023

**Published:** 2022-11-11

**Authors:** Zongwei Chen, Hong Tan, Xuemei Liu, Minghua Tang

**Affiliations:** ^1^Department of Cardiology, Affiliated Zhongshan Hospital of Dalian University, Dalian 116001, Liaoning, China; ^2^Department of Cardiology, The Second Affiliated Hospital of Dalian Medical University, Dalian, Liaoning 116023, China

## Abstract

**Objective:**

To investigate the application effect of 24 h dynamic electrocardiogram in the diagnosis of asymptomatic myocardial ischemia with arrhythmia in elderly patients with coronary heart disease.

**Methods:**

A total of 206 elderly patients suspected of coronary heart disease (CHD) with asymptomatic myocardial ischemia and arrhythmia were selected as the research subjects. 24 h dynamic electrocardiogram and conventional electrocardiogram examinations were conducted. Coronary angiography was used as the gold standard to observe the performance of the two examination methods in the diagnosis of asymptomatic myocardial ischemia with arrhythmia in elderly patients with CHD.

**Results:**

Coronary angiography showed 174 positive cases and 32 negative cases among the 206 patients. The diagnostic results of a conventional electrocardiogram showed 150 positive cases and 20 negative cases. Its sensitivity, specificity, accuracy, positive predictive value, and negative predictive value were 86.21%, 62.50%, 82.52%, 92.59%, and 45.45%, respectively. The diagnostic results of 24 h dynamic electrocardiograms showed 168 positive cases and 29 negative cases. Its sensitivity, specificity, accuracy, positive predictive value, and negative predictive value were 96.55%, 96.63%, 95.63%, 98.25%, and 82.86%, respectively. The above results indicated that 24 h dynamic electrocardiogram was significantly better (*P* < 0.05). The detection rate of arrhythmia types by 24-hour dynamic electrocardiogram was significantly higher than that of conventional electrocardiogram (*P* < 0.05).

**Conclusion:**

24 h dynamic electrocardiogram is helpful for the diagnosis of asymptomatic myocardial ischemia with arrhythmia in elderly patients with CHD and can improve the detection rate, thereby providing a basis for clinical diagnosis and treatment.

## 1. Introduction

Coronary heart disease (CHD) is a clinical coronary atherosclerotic heart disease. In general, the main pathogenesis of CHD is vascular stenosis or obstruction caused by atherosclerosis in patients, resulting in myocardial hypoxia and ischemia, so myocardial ischemia is one of the main symptoms of CHD [1]. With the gradual increase of the aging population in China, the occurrence of CHD is also becoming more and more serious, and some patients with the coronary syndrome often have arrhythmias due to ischemia manifestations. This type of patient has a risk of sudden cardiac death and myocardial infarction higher, so CHD complicated with arrhythmia has become a key issue in clinical research at this stage [2]. However, the vast majority of patients with CHD often present asymptomatic myocardial ischemia. Although such patients have obvious coronary artery occlusion, they have no angina pectoris, which may be due to the relatively slow or even slow response of elderly patients to pain. Therefore, early diagnosis and treatment are necessary to avoid delaying the disease and missing the opportunity for treatment [3]. The clinical electrocardiogram can play a good role in early diagnosis and treatment and can detect pathological *Q* waves and ST-segment elevation in time, with occasional irregular fluctuations. Therefore, it is also of great significance for clinical guidance of treatment and prognosis evaluation [4]. However, there is still controversy about the choice of diagnostic method for asymptomatic myocardial ischemia with arrhythmia in elderly patients with CHD. In view of this, this paper aims to analyze the clinical diagnostic value of 24 h dynamic electrocardiogram for asymptomatic myocardial ischemia with arrhythmia in elderly patients with CHD. The specific contents are shown as follows:

## 2. Materials and Methods

### 2.1. General Information

A total of 206 elderly patients suspected of having CHD with asymptomatic myocardial ischemia and arrhythmia were selected as the research subjects. Inclusion criteria were as follows: ① Examined by the electrocardiogram stress test, myocardial imaging, coronary angiography, and other examinations, patients met the indications of asymptomatic myocardial ischemia with arrhythmia in CHD [5]; ② patients older than 60 years; and ③ the clinical data were complete, and the patients gave informed consent. Exclusion criteria were as follows: ① Patients with severe cardiopulmonary, hepatic, and renal insufficiency; ② patients with poor compliance and were unable to cooperate with the examination; ③ patients accompanied by other cardiomyopathies; ④ patients complicated with neurological diseases; ⑤ patients with poor image quality; ⑥ patients with a history of angina pectoris. The included subjects included 113 males and 93 females, with an average age of 60–79 (65.57 ± 5.33) years, 74 patients have underlying diseases of hypertension, 67 patients have hyperlipidemia, and 65 patients have diabetes. A controlled trial study was initiated after the approval of the research ethics committee.

### 2.2. Methods

Conventional electrocardiogram: After admission, we performed an electrocardiogram examination, took the supine position, cleaned the electrode placement site and applied the special conductive paste to reduce skin resistance, connected the electrocardiogram machine to the power supply and ground wire, and the voltage was set to to 10 mm/mV, input impedance ≥100 KΩ, frequency response 100 Hz, paper feeding speed 25 mm/s, etc., adjusted the sensitivity controller, traced the conventional 12 leads, in turn, gave a clear indication of the patient's name, department, date, time, and other information. The positive diagnostic criteria of a conventional electrocardiogram are ST segment level drops in the range of 0.05∼0.2 mV, the ST segment is abnormally elevated, and the *T* wave in the same lead is smaller than the *R* wave [6].

24 h dynamic electrocardiogram: took the same supine position, the patch area should be kept clean, after connecting to the power supply and connecting the electrodes, the ST-T segment changes, duration, heart rate variability, etc. were recorded by using a BS6930 Holter electrocardiograph (Shenzhen Bosheng Medical Equipment Co., Ltd.). During the examination, cotton loose clothing should be selected as much as possible to reduce electrostatic interference; the dynamic changes of 12 leads should be traced in turn, and the patient information should be noted in detail. The positive diagnostic criteria of 24 h dynamic electrocardiogram: the ST segment is in a downward state (continuous for 0.08 s after the *J* point), the distance reaches 0.1 mV, the continuous abnormal fluctuation time is about 1 min, and the interval between two seizures is longer than 1 min [7].

### 2.3. Coronary Angiography

Coronary angiography is the gold standard for the diagnosis of CHD with arrhythmia. Before performing angiography, we performed breathing training on patients and chose the appropriate body position and angle at the same time, recorded coronary arteries, abnormal anatomy, blood flow, etc. Positive diagnostic criteria for coronary angiography: the stenosis degree of one or more coronary arteries is ≥50%, or the stenosis degree of main branch coronary arteries is ≥50%. If the above criteria are not met, the patient is negative [8].

### 2.4. Observation Indicators

We took coronary angiography as the gold standard to observe the diagnostic performance of two inspection methods, including sensitivity, specificity, accuracy, positive predictive value, and negative predictive value. Sensitivity = true positive number/(true positive number + false negative number) *∗* 100%; specificity = true negative number/(true negative number + false positive number) *∗* 100%; accuracy = (true positive number + true negative number)/total number *∗* 100%; positive predictive value = true positive number/(true positive number + false positive number) *∗* 100%; negative predictive value = true negative number/(true negative number + false negative number) *∗* 100%.

According to the electrocardiogram start and end characteristics, heart rate, rhythm, and fluctuations recorded the detection rate of arrhythmia types in the two groups, including ventricular tachycardia, ventricular arrhythmia, atrial arrhythmia, and supraventricular tachycardia.

### 2.5. Statistical Method

EXCEL spreadsheet was used for statistical analysis of experimental data, and SPSS 22.0 statistical tools were used for analysis and processing, with ($\overset{-}{x}\pm s$) for measurement, % for percentage, and *t* and *X*^2^ tests were performed respectively. *P* value < 0.05 shows that there is a significant difference between the groups.

## 3. Results

### 3.1. Diagnostic Efficacy of Conventional Electrocardiogram for Asymptomatic Myocardial Ischemia with Arrhythmia in Elderly Patients with CHD

Coronary angiography showed that among the 206 patients, 174 were positive and 32 were negative; the diagnostic results of conventional electrocardiogram showed that 150 cases were positive and 20 cases were negative, the sensitivity, specificity, accuracy, positive predictive value, and negative predictive value were 86.21%, 62.50%, 82.52%, 92.59%, and 45.45% respectively, as shown in Table 1.

### 3.2. The Diagnostic Efficacy of 24-h Dynamic Electrocardiogram in Asymptomatic Myocardial Ischemia with Arrhythmia in Elderly Patients with CHD

24 h dynamic electrocardiogram diagnosis results showed that 168 cases were positive and 29 cases were negative. The sensitivity, specificity, accuracy, positive predictive value, and negative predictive value were 96.55%, 96.63%, 95.63%, 98.25%, and 82.86%, respectively, as shown in Table 2.

### 3.3. Comparison of the Diagnostic Performance of the Two Groups of Inspection Methods

Comparing the diagnostic performance of the two groups, the diagnostic performance of 24 h dynamic electrocardiogram was significantly better than that of a conventional electrocardiogram (*P* < 0.05), as shown in Table 3.

### 3.4. Comparison of the Detection Rate of Arrhythmia Types between the Two Inspection Methods

In the 24-hour dynamic electrocardiogram test of all patients, there are four arrhythmia types including ventricular tachycardia, ventricular arrhythmia, atrial arrhythmia, and supraventricular tachycardia. The detection rate of arrhythmia types in the 24 h dynamic electrocardiogram group was 80.58% (166/206), which was significantly higher than that in the conventional electrocardiography group, which was 70.39% (145/206) (*X*^2^ = 5.784, *P* < 0.05), as shown Figure 1.

## 4. Discussion

CHD is also known as ischemic heart disease. When the continuous release of cytokines makes fibrous adipose tissue lesions and in the blood pressure, vascular branch formation and platelet aggregation, and other abnormal hemodynamic conditions, led to arterial intima, function damage, and atherosclerosis. Atherosclerosis is one of the main pathological mechanisms of CHD. Atherosclerosis and CHD are common diseases that lead to organ diseases, myocardial ischemia, and hypoxia. Relevant studies [9] have confirmed that early diagnosis and treatment are particularly important for improving the prognosis of patients with CHD. However, for patients with asymptomatic myocardial ischemia, although there is objective evidence of myocardial ischemia, there is no clinical symptom of myocardial ischemia, so even if patients frequently suffer from myocardial ischemia, the optimal time for diagnosis and treatment is still delayed because of no pain.

Coronary angiography, as the gold standard for diagnosing CHD, can quantitatively measure coronary lesions by puncturing the artery with a custom-made catheter and visualize it with a contrast agent and observe the arterial blood flow and myocardial perfusion to select an appropriate treatment method. However, coronary angiography is expensive and requires certain medical equipment and technology, so it cannot be widely used in some grass-roots hospitals and township hospitals [10]. Therefore, it is extremely important to find an effective early diagnosis method for patients.

As one of the inspection methods to reflect the bioelectric changes of human myocardial cells, electrocardiography can observe whether there is myocardial ischemia and the existence of ischemic blood vessels to diagnose the disease. However, routine electrocardiography detects the resting state of the patient, which may lead to misdiagnosis or missed diagnosis of the patient, thus affecting the follow-up treatment [11]. The emergence of dynamic electrocardiography has brought good news to patients and clinicians. As one of the clinical noninvasive diagnostic methods, it has the advantages of being affordable, it is easy to be operated, and it is noninvasive. It can continuously record the ST fluctuation trend, heart rate variability, heart rhythm, and other electrical signal data in different states within 24 hours and analyze the changes of the heart in active and resting states through 12 leads. On the one hand, it can also analyze the relationship between ST fluctuation and time, monitor the changes in patients' hemodynamics, and determine the lesion site to determine whether the patient is asymptomatic myocardial ischemia [12]. On the other hand, in the diagnosis of arrhythmia, it is possible to understand the characteristics of arrhythmia occurrence, duration, attack frequency, etc., to clarify the type of disease, to effectively improve the detection rate, to provide a scientific basis for clinical treatment and diagnosis, and to take preventive measures as soon as possible [13]. The results of this study showed that the diagnostic effect of 24 h dynamic electrocardiography was better than that of conventional electrocardiography, and the detection rate of arrhythmia types was also significantly higher than that of conventional electrocardiography, indicating that the diagnostic effect of 24 h dynamic electrocardiography was more advantageous. The reason for this may be that, compared with conventional electrocardiography, 24h electrocardiography examination can observe the nature of coronary lesions through angiography, and with the help of multi-lead synchronous, long-term and continuous monitoring of electrocardiography changes, the scope of diagnosis can be expanded, and patients' resting and active symptoms can be expanded. 24-h dynamic electrocardiography has many advantages, for example, it can record all types of arrhythmia, ST segment, *T* wave, and heart rate in detail in patients, providing important reference information for clinical diagnosis and treatment. In addition, patients can wear it tightly, which can reduce restrictions on their activities and is more acceptable to patients [14].

To sum up, 24 h dynamic electrocardiography can play a great advantage in detecting electrocardiography signals in asymptomatic myocardial ischemia with arrhythmia in elderly patients with CHD, and its diagnostic efficiency and arrhythmia detection rate is significantly higher than those of conventional electrocardiography. In addition, compared with arteriography, its detection cost and equipment requirements are relatively low and simple, and there is little difference from conventional electrocardiography. Therefore, 24-hour dynamic electrocardiography is of great significance in the early diagnosis, treatment, and prevention of patients with CHD and arrhythmia, which is worth popularizing.

## Figures and Tables

**Figure 1:** Comparison of detection rates of arrhythmia types between the two inspection methods (*n* (%)).

**Table 1:** Diagnostic efficacy of conventional electrocardiogram for asymptomatic myocardial ischemia with arrhythmia in elderly patients with CHD (*n*).

Conventional electrocardiogram	Pathological result		Total
	Positive (174 cases)	Negative (32 cases)	
Positive	150	12	162
Negative	24	20	44
Total	174	32	206

**Table 2:** The diagnostic efficacy of 24 h dynamic electrocardiogram in asymptomatic myocardial ischemia with arrhythmia in elderly patients with CHD.

24 h dynamic electrocardiogram	Pathological result		Total
	Positive (174 cases)	Negative (32 cases)	
Positive	168	3	171
Negative	6	29	35
Total	174	32	206

**Table 3:** Comparison of the diagnostic efficacy of the two groups of examination methods (*n*/*N*).

Diagnostic method	Sensitivity	Specificity	Accuracy	Positive predictive value	Negative predictive value
Conventional electrocardiogram	86.21% (150/174)	62.50% (20/32)	82.52% (170/206)	92.59% (150/162)	45.45% (20/44)
24 h dynamic electrocardiogram	96.55% (168/174)	96.63% (29/32)	95.63% (197/206)	98.25% (168/171)	82.86% (29/35)

## Data Availability

The data can be obtained from the corresponding author upon reasonable request.

## References

[1] Guangwei H., Xiyang L., Wei L. (2022). PCSK9 inhibition protects against myocardial ischemia-reperfusion injury via suppressing autophagy. *Microvascular Research*.

[2] Xia L., Dianxuan G., Ying C. (2020). Interplay of pro-inflammatory cytokines, pro-inflammatory microparticles and oxidative stress and recurrent ventricular arrhythmias in elderly patients after coronary stent implantations. *Cytokine*.

[3] Gabriele C., Claudio M., Stefano De S. (2019). Clinical impact of valvular heart disease in elderly patients admitted for acute coronary syndrome: insights from the elderly-ACS 2 study. *Canadian Journal of Cardiology*.

[4] Adyasha R., Debahuti M., Kaijian X. (2022). Improved heart disease detection from ECG signal using deep learning based ensemble model. *Sustainable Computing: Informatics and Systems*.

[5] Wenrong W., Qiang Z. (2021). Diagnostic value of scoring model of treadmill exercise test combined with dynamic electrocardiogram for latent coronary heart disease. *Journal of Electrocardiology*.

[6] Li H., Wang X., Liu C., Li P., Jiao Y. (2021). Integrating multi-domain deep features of electrocardiogram and phonocardiogram for coronary artery disease detection. *Computers in Biology and Medicine*.

[7] Ertan B., Ozal Y., Rajendra A. (2020). 1D-CADCapsNet: one dimensional deep capsule networks for coronary artery disease detection using ECG signals. *Physica Medica*.

[8] ShanWei C., Shir L., WangCan Y. (2022). Review of ECG detection and classification based on deep learning: coherent taxonomy, motivation, open challenges and recommendations. *Biomedical Signal Processing and Control*.

[9] Robert M. A., Shannon M. A. (2020). Man with dynamic ECG changes. *Annals of Emergency Medicine*.

[10] Lingxiao M., Wenjun T., Yanchun Z. (2022). Enhancing dynamic ECG heartbeat classification with lightweight transformer model. *Artificial Intelligence in Medicine*.

[11] Vafaie M. H., Ataei M., Koofigar H. (2014). Heart diseases prediction based on ECG signals’ classification using a genetic-fuzzy system and dynamical model of ECG signals. *Biomedical Signal Processing and Control*.

[12] Shanshan C., Wei H., Xingjiao G.. (2017). Heartbeat classification using projected and dynamic features of ECG signal. *Biomedical Signal Processing and Control*.

[13] Arsenos P., Gatzoulis K. A., Laina A. (2022). QT interval extracted from 30-minute short resting Holter ECG recordings predicts mortality in heart failure. *Journal of Electrocardiology*.

[14] Inigo M. (2021). A novel ECG diagnostic system for the detection of 13 different diseases. *Engineering Applications of Artificial Intelligence*.

